The article "Purification, Characterization, and Hydrolysate Analysis of Dextranase From Arthrobacter oxydans G6-4B" was retracted in 2025. Reasons: compromised peer review; a conflict of interest.

# Purification, Characterization, and Hydrolysate Analysis of Dextranase From *Arthrobacter oxydans* G6-4B

**DOI:** 10.3389/fbioe.2021.813079

**Published:** 2022-02-10

**Authors:** Nannan Liu, Peiting Li, Xiujin Dong, Yusi Lan, Linxiang Xu, Zhen Wei, Shujun Wang

**Affiliations:** ^1^ Jiangsu Key Laboratory of Marine Bioresources and Environment, Jiangsu Ocean University, Lianyungang, China; ^2^ Co-Innovation Center of Jiangsu Marine Bio-industry Technology, Jiangsu Ocean University, Lianyungang, China; ^3^ College of Food Science and Engineering, Jiangsu Ocean University, Lianyungang, China; ^4^ School of Marine Science and Fisheries, Jiangsu Ocean University, Lianyungang, China

**Keywords:** isomalto-oligosaccharides, dextran, *Arthrobacter oxydans*, hydrolysis, purification

## Abstract

Dextran has aroused increasingly more attention as the primary pollutant in sucrose production and storage. Although enzymatic hydrolysis is more efficient and environmentally friendly than physical methods, the utilization of dextranase in the sugar industry is restricted by the mismatch of reaction conditions and heterogeneity of hydrolysis products. In this research, a dextranase from *Arthrobacter oxydans* G6-4B was purified and characterized. Through anion exchange chromatography, dextranase was successfully purified up to 32.25-fold with a specific activity of 288.62 U/mg protein and a Mw of 71.12 kDa. The optimum reaction conditions were 55°C and pH 7.5, and it remained relatively stable in the range of pH 7.0–9.0 and below 60°C, while significantly inhibited by metal ions, such as Ni^+^, Cu^2+^, Zn^2+^, Fe^3+^, and Co^2+^. Noteworthily, a distinction of previous studies was that the hydrolysates of dextran were basically isomalto-triose (more than 73%) without glucose, and the type of hydrolysates tended to be relatively stable in 30 min; dextranase activity showed a great influence on hydrolysate. In conclusion, given the superior thermal stability and simplicity of hydrolysates, the dextranase in this study presented great potential in the sugar industry to remove dextran and obtain isomalto-triose.

## 1 Introduction

On the condition that internal tissue of sugar cane was damaged by mechanical cutting or burning, it was vulnerable to be infected by contaminant microorganisms, such as *Leuconostoc mesenteroides* (Jiménez, 2009). Under suitable conditions, the dextransucrase from microorganisms hydrolyzed sucrose and formed dextran. In the sugarcane industry, dextran is regarded as the most widespread contaminant indicator used for quality control purposes (Oliveira et al., 2002), which could contribute to the increasing viscosity of cane juice, affecting the settling velocity and reducing raw sugar quality (Eggleston et al., 2011). The blockage of filters caused by increasing viscosity of juice and the presence of high molecular weight (Mw) dextran cause juice spills and economic losses. It was conservatively estimated that 8.8 lb will be lost, while 0.1% increase of dextran in the juice (1,000 ppm) of sugar per ton (Jiménez, 2009). Given the economic losses of dextran to the sugar industry, much attention has been drawn to hydrolyze and remove dextran in various approaches. A wide range of previous studies suggested that the depolymerization of dextran by dextranase was evaluated as the most appropriate method compared with other physical methods with poor economic feasibility (Purushe et al., 2012; Sufiate et al., 2018a; Tanoue Batista et al., 2021). Consequently, with the rapid development of protein spatial structure analysis (Chew et al., 2019; Sankaran et al., 2019; Krishna Koyande et al., 2020; Wang et al., 2022), it is a burning problem to explore the enzymatic properties and application suitable for sugar processing of dextranase.

Dextran is a macromolecular polymer (10^5^–10^7^ Da) composed of glucosaccharides linked mainly by *α*-1,6-glycoside bonds, frequently synthesized from sucrose by contaminant microorganisms (Martínez et al., 2021; Tanoue Batista et al., 2021). Dextranase (EC 3.2.1.11) catalyzes the hydrolysis of *α*-1,6-glycoside bond in dextran and cleave dextran into lower Mw fractions, isomalto-oligosaccharides (IMOs), or glucose (Khalikova et al., 2005; Zohra et al., 2015; Ren et al., 2018). In the same enzymatic hydrolysis system, a massive number of hydrolysates are present simultaneously, for instance, different Mw IMOs and dextran (Park et al., 2012; Zohra et al., 2015; Münkel and Wefers, 2019). Intriguingly, the degree of polymerization of effective oligosaccharides from 2 to 10 monosaccharide units imply multiple applications and highly commercial interest in the food and health market (Seo et al., 2007). As a non-digestible food, IMOs are beneficial to reduce the risk of cancer, obesity, and type Ⅱ diabetes (Huang et al., 2020). Based primarily on extensive literature, the sources of dextranase are diverse, including bacteria [*Streptococcus mutans* (Suzuki et al., 2012) and *Bacteroides thetaiotaomicron* (Pittrof et al., 2021)], yeast [*Lipomyces starkeyi* (Chen et al., 2008)], and fungi [*Chaetomium gracile* (Zhao et al., 2021), *Penicillium funiculosum* (Volkov et al., 2019), and *Aspergillus allahabadii* (Netsopa et al., 2019)]. Depending on the spatial structure and catalytic characteristics, dextranase can be basically categorized into GH49 and GH66 families (Ren et al., 2019). Currently, isolation and purification of dextranase from extracellular products of microorganisms, such as *Catenovulum* (Ren et al., 2018), *Streptococcus* (Suzuki et al., 2012), and *Arthrobacte*r (Ren et al., 2019), have made considerable progress in unraveling enzymology properties. Despite these advances, it has continued to be a significant challenge to address the limitation of low thermal stability and hydrolysates with irregular percentages for application. Most dextranase have been reported to maintain relatively high thermal stability below 50°C (Cai et al., 2014; Jiao et al., 2014; Wang et al., 2014; Sufiate et al., 2018b; Lai et al., 2019), even lower. Furthermore, it brings complicated steps for subsequent purification of hydrolysis products, involving glucose to IMOs even low Mw dextran with different percentages (Goulas et al., 2004; Ren et al., 2018; Abraham et al., 2019; Lai et al., 2019).

However, previous research suggested that it was challenging to control the Mw of hydrolysates synthesized by dextranase (Huang et al., 2020). In addition, industrial utilization of dextranase has been constrained by the adaptation of reaction conditions to sugar processing. Therefore, it is an efficient idea to exploit suitable dextranase in decreasing the viscosity of sugar cane juice and obtain IMOs with prebiotic functions in this study.

In order to overcome the dextran in sugarcane juice and harvest prebiotic functional products, the exploitation of dextranase with high thermal stability and hydrolysates of relatively concentrated Mw remained the objectives of the present work. In this research, a marine bacterium producing dextranase was screened, and the enzymatic characterization and protein structure were analyzed. Different hydrolyzing strategies were implemented to observe the types and proportions of hydrolytic products. The results provided new insights into the application of dextranase in the sugar industry.

## 2 Materials and Methods

### 2.1 Materials and Chemicals

The dextran (T20, T40, and T70) and agarose (sepharose) used in this study were of analytical pure grade and purchased from GE Healthcare. Oligosaccharide standard and Coomassie brilliant blue R250 and G250 were available from Sigma-Aldrich. All other reagents were of analytical grade and obtained from Sinopharm Chemical Reagent Corporation (Shanghai, China).

### 2.2 Isolation and Identification of Strains

In the course of this experiment, samples played a significant role. Samples collected from Gaogong Island were diluted with appropriate concentration and then spread on 2216E medium (Solarbio, China) containing Dextran blue 2000, cultured at 30°C for 48–72 h. The main focus of this step was to select strains with large transparent zone for further purification and enzyme activity determination. Afterward, the best dextranase-producing strain G6-4B was characterized by researching the biochemical and morphological characters. Genomic DNA was extracted, and 16S rDNA was amplified by PCR using universal primers (27F 5′-AGAGTTTGATCCTGGCTCAG-3′/1492R 5′-GGT​TAC​CTT​GTT​ACG​CTT-3′). The amplified product was purified by PCR purification kit (Bioneer, USA), and nucleotide sequencing was blasted in NCBI (https://www.ncbi.nlm.nih.gov/). MEGA 6.0 software was used to make multiple comparisons with other strains of similar genetic relationships, and neighbor-joining method was taken to build a phylogenetic tree.

### 2.3 Analysis of Protein Sequence and Structure

The composition and spatial structure of amino acids dominate most of the properties of enzymes, so the comparative analysis with other dextranase previously reported was executed. Dextranase sequence was searched from the whole-genome sequence annotations, then blasted in NCBI. Signal peptides, isoelectric points, and protein molecules were projected by SignalP-5.0 Server (http://www.cbs.dtu.dk/services/SignalP/) and ExPASy (https://prosite.expasy.org/). The 3D structure of protein was predicted by the Swiss model (https://swissmodel.expasy.org/).

### 2.4 Dextranase Production

The strain G6-4B was inoculated into the medium containing 5 g/L of peptone, 1 g/L of yeast extract, 10 g/L of dextran T20, and 10 g/L of NaCl with pH 7.5. The fermentation supernatant was collected by centrifugation (Multifuge X3R, Thermo Fisher) as crude enzyme liquid after 30 h cultivation at 30°C, 180 rpm.

### 2.5 Purification of Dextranase

Ammonium sulfate was gradually (increasing by 10%) added to the crude enzyme solution, kept at 4°C, and placed on a magnetic stirrer to ensure complete dissolution. The dextranase activity and total protein content in both precipitation and supernatant with different concentrations of ammonium sulfate were measured to confirm the most suitable concentration. Then the activity of dextranase in the precipitate was maximized for 8 h, 4°C at the most suitable concentration. Precipitated protein was obtained by centrifugation at 12,000 × *g*, 4°C for 10 min, then dissolved and dialyzed in 10 mM Tris-HCl buffer (pH 7.5). Subsequently, Millipore Centrifugal Filter Units (4 ml, 10 kD) were used for ultrafiltration of dextranase and centrifuged at 3,500 × *g*, 4°C until to a required volume. Then 200 μl of dextranase ultrafiltrated was loaded on Q Sepharose Fast Flow (1.6 cm × 10 cm, GE Healthcare, Sweden), and purification analysis was performed in AKTA pure L1 system (GE Healthcare, Sweden). The chromatography column was equilibrated by 50 mM Tris-HCl (pH 7.5) before loading. Gradient elution was carried out with 1 M NaCl at a flow rate of 1 ml/min for 10 min and collected by an automatic fraction collector. The dextranase activity and protein content in each collecting tube were determined, then the separation enzyme was ultrafiltrated by Millipore Centrifugal Filter Units (4 ml, 10 kD). All of the above were designed to acquire approximately purified dextranase.

### 2.6 Dextranase Characterization

#### 2.6.1 Effects of Temperature and pH on Dextranase Activity and Stability

In this experiment, various temperatures and pH were set to investigate the essential character of dextranase. The activity of dextranase was determined at different reaction temperatures (40°C–70°C) and diverse pH (4.0–9.0), respectively. Incubated at 40, 50, and 60°C for 0–5 h, the thermal stability was evaluated by measuring the dextranase activity at each interval. Analogously, the pH values of the enzyme solution were adjusted to 4.0–9.0 by various buffer solutions, then the residual activities were determined under the optimum condition after 1 h cultivation. Buffer systems were based on previous experiments (Ren et al., 2018; Lai et al., 2019), including 50 mM acetic acid-sodium acetate buffer (pH 4.0–5.5), 50 mM sodium phosphate buffer (pH 5.5–7.5), and 50 mM Tris-HCl (pH 7.5–9.0).

#### 2.6.2 Effects of Metal Ions on Dextranase Activity

The enzyme solution was mixed with a series of metal ions at 55°C, and the final concentration of metal ions reached 1, 5, and 10 mM by appropriate dilution. Relative enzyme activity was determined by percentage conversion with the enzyme activity without metal ions as the control after 30 min.

### 2.7 Hydrolysate Analysis

In preliminary experiments, estimated different enzymatic hydrolysis systems were estimated: hydrolysis of 3% T20, T40, and T70 for 1 h (3 U/ml), hydrolysis of 3% T20 for 30 min, 1 and 3 h (3 U/ml), and 0.5% T20 hydrolyzed by different concentrations of dextranase (0.5, 1, and 5 U/ml) for half an hour. All the above reactions were implemented at 55°C and pH 7.5. Finally, hydrolysates were filtered by a 0.22-μm membrane and subjected to HPLC and LC-MS. The products were detected and analyzed by Waters Sugar-Pak1 (300 mm × 7.8 mm; Milford, United States) HPLC with a differential refraction detector. Methods of HPLC were based on previous experiments (Ren et al., 2018). In order to further identify the hydrolysates, LC-MS was performed. The liquid chromatography was Agilent 1100 Series LC Chem Station and analyzed by Zorbax SB-C_18_ (5 μm, 0.5 mm × 250 mm, Agilent Technologies, United States). The mobile phase was 15 mM PTA acetonitrile solution (70%, pH 7.0) at 10 μl/min, the column temperature was adjusted to 35°C, and the injection volume was 2 µl. ESI-IT-TOF (SHIMADZU, JAPAN) high-resolution tandem resolution mass spectrometry was used for detection under the following conditions: in positive ion mode, the spray voltage and current were 3.6 kV, and 0.5 L/min, respectively; the ion source temperature was 200°C, the detection voltage was 1.8 kV.

## 3 Result

### 3.1 Isolation and Identification of Dextranase-Producing Strain

The strain G6-4B (Figure 1) illustrated the highest dextranase-producing ability according to the size of clear zone. Based on the sequence alignment of 16S rDNA and the construction of a phylogenetic tree (Figure 2), strain G6-4B was characterized as *Arthrobacter oxydans* (accession number OL377850). The 16S rDNA sequence was compared with other related species sequences by BLAST, and the greatest similarity with *Arthrobacter oxydans* was revealed*.*

**FIGURE 1:** Transparent zone formed by G6-4B on the plate containing blue dextran **(A)** and scanning electron micrograph **(B)**.

**FIGURE 2:** Phylogenetic tree based on 16S rDNA gene sequences.

### 3.2 Structural Characteristics of Dextranase

The amino acid sequence-encoded dextranase potentially was searched in annotation information for complete genome sequencing of G6-4B and identified as dextranase of the GH49 family by comparison in the NCBI (accession number OL439772). A total of 640 amino acids with a predicted Mw of 71.12 kDa were consistent with the result of SDS-PAGE gel, which followed. As expected, the isoelectric point was forecast to be 4.8, and there were four glycosylation sites in the total sequence. The SignalP-5.0 indicated that a 32-amino acid signal peptide at the N-terminal belongs to SPⅠ. Swiss model prediction results showed that the sequence identity with dextranase (6nzs.1. A) from *Arthrobacter oxydans* KQ11 was 88.74%. In correspondence with dextranase of GH49, the dextranase in this study was partitioned into two main domains: the N-terminal domain was identified as a *β* sandwich composed of 190 amino acids, and the other domain was a right-handed parallel *β*-helix consisting of three parallel sheets at C-terminal (Larsson et al., 2003). *β*-helix is one type of *β*-solenoids and provides a large elongated surface to accommodate multiple binding sites when combining with flexible molecules, such as carbohydrates (Kajava and Steven, 2006). All structural characteristics above were favorable for combination with dextran and hydrolysis reaction.

### 3.3 Purification and Characterization of Dextranase

#### 3.3.1 Ammonium Sulfate Precipitation

Ammonium sulfate gradients increasing experiment displayed that 70% ammonium sulfate could precipitate the maximum dextranase proteins from fermentation supernatant. Compared with the crude enzyme solution, dextranase was purified 7.40-fold with a specific activity of 66.26 U/mg protein and a yield of 46.62% Table 1. The optimal concentration of ammonium sulfate and enzyme activity precipitated are discrepants closely linked to the source of dextranase.

**TABLE 1:** Purification of dextranase from G6-4B

Purification Step	Total activity (U) (mg)	Table protein (mg)	Specific activity (U/mg)	Purification (Fold)	Yield (%)
Culture	3103.73	346.40	8.96	1	100
Ammonium sulfate precipitatio	1446.96	21.84	66.26	7.40	46.62
Ultrafiltration	1215.11	7.94	153.04	17.08	39.15
Anion exchange chromatograph	337.69	1.17	288.62	32.25	10.88

#### 3.3.2 Ultrafiltration

The ultrafiltration of dextranase was treated with Millipore Centrifugal Filter Units (10 kD) to remove other low-Mw interfering proteins. Through a filter, about 7.47% of dextranase activity was lost, and specific enzyme activity was enhanced to 153.04 U/mg of protein.

#### 3.3.3 Anion Exchange Chromatography

In line with the isoelectric point of dextranase, anion exchange chromatography was adopted in order to optimize the purification. Dextranase was successfully purified up to 32.25-fold with a specific activity of 288.62 U/mg of protein and retained 10.88%. Finally, it was issued as a single band of an estimated Mw of 70 kDa in SDS-PAGE gel, which was supported by the results of the predicted SignalP-5.0 (Figure 3).

**FIGURE 3:** Sodium dodecyl sulfate-polyacrylamide gel electrophoresis (SDS-PAGE) of dextranase from G6-4B. M, protein marker; Lane 1, purified dextranase.

#### 3.3.4 Effects of Temperature and pH on Dextranase Activity and Stability

Dextranase from G6-4B performed a comparatively higher activity in 40°C–60°C (Figure 4A); 55°C was the optimum temperature upon further experimentation. Above 70°C, nearly 66% of the enzyme activity (190.49 U/mg) was significantly lost compared with the optimal temperature. The thermal stability diagram suggested that the dextranase activity remained at least 93% (268.42 U/mg) for 3 h at 50°C, and nearly 60% (173.17 U/mg) was maintained following storage at 60°C for 5 h (Figure 4C). Figures 4B,D showed the effects of pH on dextranase activity and stability. It appeared that the highest activity was at pH 7.5, and the relatively high level remained in the range of pH 7.0–9.0, which was consistent with the pH of sugarcane juice increasing above 7.0 during the sugar manufacturing process (Jiménez, 2009). However, under acidic conditions (at pH 3.0–6.0), more than 50% of the enzyme activity was lost. In general, dextranases from strain G6-4B could maintain a relatively high level in neutral to alkalescent environment.

**FIGURE 4:** Effects of temperature **(A)** and pH **(B)** on dextranase activity and stability **(C)** and **(D)**.

#### 3.3.5 Effects of Metal Ions on Dextranase Activity

Certain metal ions like Ca^2+^, Mn^2+^, and Mg^2+^, which were reported to exist in sugarcane juice, were required for alkaline protease highest activity (Ma et al., 2007). Table 2 indicated the efforts of various metal ions with three concentrations (1, 5, and 10 mM) of dextranase activity. Ba^2+^, Ca^2+^, and Mg^2+^ showed less than 40% inhibiting effects to dextranase activity while the dextranase activity was completely inhibited when Ni^+^, Cu^2+^, Zn^2+^, Fe^3+^, and Co^2+^presented in the buffer, even at low concentrations (1 mM). Several metal ions, such as Mn^2+^, Na^+^, K^+^, and NH_4_^+^ showed higher inhibition with the increase of ions concentration (10 mM). No metal ions were discovered to increase the dextranase activity, which was opposite to the report of dextranase from *Hypocrea lixii* F1002 (Wu et al., 2011). Future studies could fruitfully explore this issue further by genetic modification or other means to match the requirements of the sugar industry.

**TABLE 2:** Inhibition of metal ions to dextranase

Compound	Relative activity(%)	Relative activity(%)	Relative activity(%)
	1 mM	5 mM	10 mM
Control	101.13 ± 3.79	103.53±5.28	104.27 ± 4.03
Si^2+^	64.23 ± 3.08	62.29±2.84	59.17 ± 2.73
Mn^2+^	61.51 ± 5.32	40.99±3.18	23.30 ± 1.85
Mg^2+^	76.57 ± 4.03	72.49±3.71	61.61 ± 2.83
Co^2+^	5.22 ± 0.64	0	0
Na^+^	65.30 ± 5.19	55.77±4.80	41.29 ± 3.55
Ni^+^	0	0	0
Cu^2+^	0	0	0
Ba^2+^	75.02 ± 4.28	68.80 ± 5.02	69.09 ± 2.76
Ca^2+^	72.10 ± 4.16	64.91 ± 3.64	61.22 ± 1.81
Li^+^	59.08 ± 3.08	54.21 ± 4.11	54.60 ± 1.64
Zn^2+^	0	0	0
K^+^	65.20 ± 2.86	60.73 ± 3.74	38.47 ± 0.59
Fe^3+^	0	0	0
NH_4_^+^	55.67 ± 4.73	44.10 ± 2.52	34.19 ± 2.07

### 3.4 Analysis of End Products of Different Hydrolysis Systems

More generally, dextranase could degrade high-Mw dextran to oligosaccharides with different degrees of polymerization or low Mw dextran by hydrolysis of *α*-1,6 glycoside bond (Gan et al., 2014). Especially, the Mw of dextran, dextranase activity, and hydrolysis time are very sensitive to the degree of hydrolysate polymerization. Figure 5 and Table 3 display the HPLC and LC-MS results of the principal products released by dextranase from G6-4B in different hydrolysis systems. What is noteworthy in this study was that the types of end products of hydrolyzing different Mw dextrans (T20, T40, and T70) were mainly isomalto-triose; the polymerization of hydrolysates did not affiliate with the reaction time markedly after 30 min. On the other hand, dextranase activity had a great influence on the type of hydrolysates.

**TABLE 3:** LC-MS results of hydrolysates by dextranase

Compound	Mass	Abund	Relative amount
C_18_H_32_O_16_	504.17	4802	73.19%
C_24_H_42_O_21_	666.22	760	11.58%
C_36_H_62_O_31_	990.33	527	8.03%
C_42_H_72_O_36_	1152.38	472	7.19%

**FIGURE 5:** Hydrolysates of different hydrolysis systems by HPLC. **(A)** standards from G1 to G7 were glucose, maltose, isomalto-triose, isomalto-tetraose, isomalto-pentaose, isomalto-hexaose, and isomalto-heptaose, respectively. **(B)** Hydrolysates of 3% T20, 3%T40, and 3%T70 after 1 h. **(C)** Hydrolysates of 3% T20 after 30 min, 1 h, and 3 h. **(D)** Hydrolysates of 0.5%T20 by different dextranase activity (0.5, 1, and 5 U/ml).

#### 3.4.1 Influence of the Degree of Dextran Polymerization on Final Products

Investigations on the hydrolysis of dextran with varying Mw were a sign of the progress of decomposition changes when starting from the disparate initial Mw, especially in lower enzyme levels (Abraham et al., 2019). Consequently, the effects of dextran polymerization on the type of hydrolytic products by dextranase from G6-4B were first investigated in this study. More than 70% of the hydrolysates in 30 min were G3 and G4, with a small amount of dextran substrate (3% T20, 3% T40, and 3% T70), which were not completely hydrolyzed, as evidenced by HPLC results (Figure 5B). However, hydrolysis of dextran from T20 to T70 did not yield glucose or medium Mw dextran. This characteristic of dextranase creates significant superiority in the production of oligosaccharides with a certain degree of polymerization.

#### 3.4.2 Effect of Reaction Time on the Final Products

Generally, the Mw of decomposition products decreased with the increase in incubation time following a gradual pattern (Abraham et al., 2019). Moreover, the proportion of hydrolysates varied with the extension of incubation time. Figure 5C shows the hydrolysates at different incubation times. After 30 min of hydrolysis, more than 70% of dextran was completely hydrolyzed to oligosaccharides (G3 accounted for more than 70%, and the rest was mainly G4). When the incubation time was extended from 30 min to 3 h, the types of hydrolysates did not change significantly.

#### 3.4.3 Effect of Enzyme Activity on End Products

The results were summarized in Figure 5D, reflecting that the increases in dextranase activity resulted in hydrolysates of different components gradually becoming simple (incubation for 30 min), indicating that the concentration of dextranase was the key factor determining hydrolysates. Residual dextran and oligosaccharides (G7, G4, and G3) remained coexisting at an activity of 0.5 U/ml. When enzyme activity increased to 1 U/ml, the content of residual dextran decreased gradually, while the content of oligosaccharides (G6, G4, and G3) accumulated. Finally, species of hydrolysates (principally G3 and G4) remained stable at 5 U/ml; increasing more activity did not affect hydrolysates.

#### 3.4.4 LC-MS Analysis of End Products

Considering that the Mw of dextran synthesized by contaminant microorganisms kept a general concentration of 0.1%–0.5% (Abraham et al., 2019), the hydrolysates of 0.5% T20 for 30 min were selected for LC-MS. Table 3 reveals that the major hydrolysates were isomalto-triose, accounting for 73.19%, and the rest were isomalto-tetraose (11.58%), isomalto-hexaose (8.03%), and isomalto-heptaose (7.19%). Depending on the above data, the possibility of controlling the types of hydrolysates could be realized by regulating the activity level of dextranase, especially to obtain isomalto-triose.

## 4 Discussion

According to previous reports, the sources of dextranase were extensive, ranging from ocean, soil, and the tissues of diverse plants. Consistent with G6-4B in this research, dextranase production strains, such as *A. oxydans* KQ11 (Wang et al., 2014) and *Catenovulum* sp. DP03 (Cai et al., 2014) reported, were both derived from the marine environment. Dextranase from various microbial sources showed discrepant structures, and the Mw tended to be concentrated at 40–140 kDa, although there were exceptions. The Mw of dextranase from *Penicillium lilacinum* (Das and Dutta, 1996) was only 26 kDa, while the Mw of dextranase from *Bacillus licheniformis* KIBGE-IB25 (Zohra et al., 2015) was large up to 158 kDa. The Mw of dextranase from G6-4B was analogous to the dextranase from *C. gracile* (71 and 77 kDa), which were commercially used for dextran removal in the sugar industry (Khalikova et al., 2005). Additionally, in the light of the crystal structure of dextranase protein published in Protein Date Bank (PDB), the Mw of dextranase in GH66 (3VMN, 5AXG) was generally higher than that of GH49 (6NZS, 1OGO). It was conjectured that the differences were attributed to various domain compositions of the two families.

High thermal stability is one of the preconditions for dextranase application in the sugar industry. Previous results (Cai et al., 2014; Jiao et al., 2014; Wang et al., 2014; Sufiate et al., 2018b; Lai et al., 2019) had shown that the optimum reaction temperature of dextranase mostly ranged from 25°C to 60°C, which was possibly related to the physiological characteristics and survival environment of various strains. In general, the rate of chemical reaction increases with high temperature. However, as a protein, when the temperature is exorbitant, the enzyme protein will be irreversibly deformed, resulting in the enzyme losing catalytic activity. Similarly, within a certain pH range, the enzyme shows catalytic activity, but beyond the pH range, the enzyme activity will fade or even lose. Deng et al. (2020) reported that the expression of dextranase from marine bacteria in *Escherichia coli* showed no activity at 50°C for 1 h. On the contrary, a thermostable dextranase isolated from the Great Artesian Basin of Australia exhibited optimum activity at 70°C (Wynter et al., 1996). In order to neutralize more acid pH values produced by juice derived from the deteriorated sugar cane, large amounts of lime were consumed. So, the pH values of juice varied from acidic (pH 5.5–6.0) to neutral or slightly alkaline (pH 7.0–8.0), with a relatively wide range. At the stage of juice clarification, the temperature was generally up to 65°C or higher (Jiménez, 2009). Compared with dextranase from the majority strains, dextranase in this study has greatly improved the tolerance to high temperature; such characteristics were more adaptable for the application of high-temperature sugar milling processes in the sugarcane industry. Nevertheless, the performance of pH and metal ion stability was not satisfactory (Lee et al., 2017; Phong et al., 2018). Relatively high enzyme activity could be maintained only in neutral to slightly alkaline environment, distinguished from the dextranase from *Streptomyces* sp. NK458 (Purushe et al., 2012) and *Chaetomium gracile* (Zhao et al., 2021), which displayed high enzyme activity ranging from pH 5.0 to 10.0 (>50% activity). Certain metal ions exhibited to promote dextranase activity, for example, Fe^2+^ and Li^+^ (Huang et al., 2019). Moreover, contrary to the results of our study, the existence of Co^2+^, Mn^2+^, Ca^2+^ accelerated the activity of dextranase from *A. allahabadii* X26 (Netsopa et al., 2019). Therefore, the stability still needs to be further improved to better adapt to industrial applications.

The main hydrolysates of different Mw dextran were all isomalto-triose, accompanied by a small amount of isomalto-tetraose, isomalto-hexaose, and isomalto-heptaose. The species of hydrolysates were greatly affected by dextranase activity, did not change with time extension after 30 min of reaction. Compared with the dextranase from *H. lixii* F1002 (Gan et al., 2014), which obtained a series of dextran with decreasing Mw within 90 min, the dextranase in this study reflected a distinct hydrolysis process. The species of hydrolysates were significantly different from most reported dextranase, which hydrolysates was relatively dispersed, including glucose (Lai et al., 2019), maltose (Lai et al., 2019), isomalto-triose (Ren et al., 2018), to dextran of medium Mw (Abraham et al., 2019). In addition, this reaction pattern was significantly different from the previously reported hydrolysis trend of dextranase (Deng et al., 2020), in which, the proportion of hydrolysates varied from 0.5 to 6 h. These phenomena indicated that the dextranase in this study was suitable for the application in the sugar industry, which was largely realized within the first 30 min of incubation time. Based on the catalytic properties of dextranase, the production of IMOs with specific Mw by dextranase has been developed by immobilization technology or the construction of multiple enzymatic reaction systems. For example, the formation ratio of IMOs with specific Mw was controlled by establishing a double enzyme reaction system of dextranase and dextransucrose maltose acceptor reaction (Huang et al., 2020). IMOs with polymerization degree of 8–10 could be quantitatively produced by immobilizing dextranase on epoxy-activated global convective interaction medium (CIM^®^) disk and adjusting the amount of immobilized enzyme, substrate concentration, and flow rate (Bertrand et al., 2014). Future studies could conduct an inquiry into the association between hydrolysates with dextranase and pay attention to more efficient development and utilization of dextranase.

## 5 Conclusion

The dextranase-producing strain *Arthrobacter oxydans* G6-4B was isolated and identified from Gaogong island. The dextranase was successfully purified up to 32.25-fold with a specific activity of 288.62 U/mg protein. A total of 640 amino acids encoded dextranase with a Mw of 71.12 kDa and belonging to the GH49 family. The pH and temperature optima were around 7.5 and 55°C, respectively. The types of products obtained by hydrolysis of dextran with different Mw (T20, T40, and T70) were relatively consistent; isomalto-triose accounted for more than 73%, without glucose and maltose. Given its superior thermal stability and relative simplicity of hydrolysates, the dextranase in this study presented great potential in the sugar industry to remove dextran and obtain iso-maltose with prebiotic effects. Even if many unknown factors determine the hydrolysates of dextranase, our research has bridged the gap between theory and application.

## Data Availability

The original contributions presented in the study are included in the article/Supplementary Material, further inquiries can be directed to the corresponding author.
